This article has been retracted.

# Analysis on Influencing Factors of Recurrence after Indirect Inguinal Hernia Laparoscopic Surgery

**DOI:** 10.1155/2022/2978745

**Published:** 2022-01-12

**Authors:** Yuan Cao, Zhaozheng Ding, Hongjia Qiang

**Affiliations:** The First People's Hospital of LianYunGang (Pediatric Surgery), Lianyungang 222000, Jiangsu, China

## Abstract

This paper aims to analyze the recurrence of indirect inguinal hernia in children after laparoscopic surgery and investigate the influencing factors that may lead to recurrence so as to guide the prevention and treatment of postoperative recurrence of this kind of disease in the future. The data of 260 children with indirect inguinal hernia treated by laparoscopic surgery and followed up in our hospital from July 2019 to July 2021 were selected. A self-designed questionnaire was used to collect the basic data. The recurrence was analyzed, and the influencing factors of recurrence were analyzed by univariate analysis and multivariate analysis. Among 400 children after indirect inguinal hernia laparoscopic surgery, an occurrence was observed in 15 children, and the recurrence rate was 5.77%. Univariate analysis showed that the age and course of disease were not correlated with recurrence after indirect inguinal hernia laparoscopic surgery (*P* > 0.05). Being male, bilateral lesions, exact high ligation, loose hernia back wall peritoneum, deciduous ligature, incorrect ligation of the fascia of musculus obliquus externus abdominis, large inguinal hernia, circumferential wiring, and too early off-bed activity were the influencing factors of recurrence after indirect inguinal hernia laparoscopic surgery (*P* < 0.05). Logistic multivariate regression analysis showed that being male, bilateral lesions, loose hernia back wall peritoneum, deciduous ligature, incorrect ligation of the fascia of musculus obliquus externus abdominis, large inguinal hernia, and too early off-bed activity were the influencing factors of recurrence after indirect inguinal hernia laparoscopic surgery (OR>1, *P* < 0.05). Exact high ligation and circumferential wiring were protective factors of recurrence after indirect inguinal hernia laparoscopic surgery (OR>1, *P* < 0.05). After indirect inguinal hernia laparoscopic surgery, recurrences were affected by many factors, such as gender, site of pathological changes, and loose hernia back wall peritoneum. For these children with risk factors, reasonable intervention should be taken to reduce recurrence; exact high ligation and circumferential wiring are the protective factors. If permitted, the children meeting related indications can be treated by high ligation or circumferential wiring to reduce the risk of recurrence after indirect inguinal hernia laparoscopic surgery.

## 1. Introduction

Indirect inguinal hernia is common in pediatrics, and most of them are treated with surgery. Due to the application of modern minimally invasive techniques, the surgical technique continues to mature, so the overall benefit is good [1]. At present, the main minimally invasive surgery for inguinal hernia is laparoscopic surgery. This type of technology can control the incision in the range of 0.3 to 0.5 cm. Laparoscopic surgery has the advantages of less trauma, light postoperative pain, and concealed incision. It is accepted and recognized by the majority of medical workers and their families [2, 3]. However, for some complex inguinal hernias, including giant hernias, and incarcerated hernias, there is still a risk of recurrence after minimally invasive surgery. After recurrence, the children may need to undergo a second operation, which will bring physical and psychological consequences to them. Not only that, but it will also cause psychological and economic pressure on the parents of children [4, 5]. Therefore, early identification of the risk factors that may lead to the recurrence of children with indirect inguinal hernia after laparoscopic surgery and timely formulation and implementation of intervention strategies for the factors are of great significance to reducing recurrence. At present, there are many related studies on the factors affecting the recurrence of children with an indirect inguinal hernia. However, due to the complex recurrence mechanism of this type of disease, a unified view has not yet been formed. In order to guide the prediction and evaluation of the risk of recurrence of children with indirect inguinal hernia after laparoscopic surgery and the formulation of intervention plans, this study collected the medical records of 400 children with an indirect inguinal hernia who completed treatment and follow-up in our hospital, and this study aimed to analyze the operation of the children, including the influencing factors for later recurrence. The results are reported as follows.

## 2. Materials and Methods

### 2.1. Subject

The medical records of 400 children with an indirect inguinal hernia who completed transumbilical single-site laparoscopic surgery and postoperative follow-up in our hospital from July 2019 to July 2021 were selected, including 270 males and 130 females; 8 months to 14 years old, with an average of (6.58 ± 3.25) years old; the course of illness ranged from 1 week to 39 months, with an average of (22.73 ± 5.28) months.

### 2.2. Inclusion Criteria and Exclusion Criteria

Inclusion criteria were (1) combined with symptoms of abdominal pain and vomiting; (2) in accordance with the “Clinical Diagnosis and Treatment Guidelines-Pediatric Surgery Fascicle” [6] indirect inguinal hernia related diagnostic criteria and confirmed by B-ultrasound combined with the physical signs of the child; (3) all First onset; (4) complete medical record data; and (5) complete follow-up data. Exclusion criteria were (1) patients with trauma or tumor in the groin area; (2) patients with cirrhosis and asides; and (3) patients who received relevant treatment one month before enrollment.

### 2.3. Method

#### 2.3.1. Transumbilical Single-Site Laparoscopic Surgery

Children are instructed to empty their urine before laparoscopic surgery through a single part of the umbilical cord, and the skin is prepared on the day of surgery. General anesthesia is performed, and the child is placed in a supine position with head down and feet high. A 5 mm incision was made longitudinally on the right side of the umbilicus; subcutaneous and peritoneum were cut; a 5 mm high-definition laparoscope was inserted to establish a carbon dioxide pneumoperitoneum (pressure 10–12 mmHg); a 3 mm hole was made at the left edge of the umbilicus, and 3 mm bowel forceps or separation forceps was used. A 2 mm incision was made at the projection of the body surface of the inner ring mouth. The hernia sac was found under laparoscopy, and the hernia sac was dissociated from the high position to the inner and extraperitoneal fat plane. Some children use special hernia needles to pierce the 3–0 Vicryl absorbable thread, ligate and sew the hernia sac through the same outlet, tie the knot outside the peritoneum, and sew and close the inner ring opening. Some children use special hernia needles to pierce the 2–0 escort help line, pass under the peritoneum inside the inner ring orifice, pass through the same exit, tie a knot outside the peritoneum, and circulate the inner ring orifice. For children with incarcerated hernias, manual reduction must be performed before surgery.

#### 2.3.2. Data Collection

A self-made questionnaire of our hospital was used to collect baseline data of children. The Kronbach coefficient was 0.837, and the content included (1) age: divided into <5 years old, 6–10 years old, and >10 years old; (2) gender: divided into male and female; (3) course of disease: divided into <1 year and ≥1 year; (4) location of disease: divided into unilateral disease and bilateral disease; (5) whether the high ligation is exact during the operation: evaluate whether the hernia sac is free to the extraperitoneal fat plane by B-ultrasound; loss of continuity and integrity between the peritoneum and loose structure; (6) whether the hernia sac ligation line falls off: observe and record by the nursing staff; (7) whether the external oblique muscle fascia is misligated: after the B-ultrasound assessment, the outside of the abdomen can be seen, the oblique muscle fascia and the hernia sac are ligated together, the hernia sac is empty, or the hernia sac is not ligated, the omental structure or intestinal structure can be explored, and the abdominal and external oblique muscle fascia is displaced; (8) whether it is a huge hernia: passed B-ultrasound evaluation, finger abdominal wall defect >10 cm; (9) suturing or cerclage: recorded by the doctor who performed the operation; and (10) premature getting out of bed after the operation: recording the time of the child getting out of bed, and the child less than 2 days is counted as get out of bed prematurely.

#### 2.3.3. Evaluation Method for Postoperative Recurrence of Indirect Inguinal Hernia

Six months after the operation, the main signs and manifestations of the postoperative B-ultrasound were reviewed and combined with the diagnostic criteria in the “Clinical Diagnosis and Treatment Guidelines-Pediatric Internal Medicine” [6].

### 2.4. Statistical Analysis

SPSS 24.0 was used to process the data, the count data were expressed as %, and the comparison was performed by the *χ*2 test. The multifactor analysis of the influencing factors for the recurrence of indirect inguinal hernia in children was tested by logistic regression analysis. *P* < 0.05 indicated that the difference was statistically significant.

## 3. Results

### 3.1. Recurrence Rate

400 children with indirect inguinal hernia were followed up for 6 months after single-site laparoscopic surgery on the umbilical cord. It was found that 15 cases had recurrence after surgery, with a recurrence rate of 5.75% (23/400). According to postoperative recurrence, children were divided into recurrence group (*n* = 23) and nonrecurrence group (*n* = 377).

### 3.2. Single Factor Analysis of the Recurrence of Children with Indirect Inguinal Hernia after Surgery

The preliminary univariate test results showed that the age and course of disease were not related to the recurrence of children with an indirect inguinal hernia after laparoscopic single-site laparoscopic surgery (*P* > 0.05); male, bilateral onset, exact high ligation, posterior hernia wall peritoneum laxity, loss of hernial sac ligation line, the misligation of external oblique muscle fascia, huge hernia, cerclage, and premature getting out of bed after operation may all be the influencing factors of postoperative recurrence (*P* < 0.05). The results are shown in Tables 1 and 2.

### 3.3. Multivariate Logistic Regression Analysis

The variables preliminarily confirmed as influencing factors by the single factor test were included and assigned, including gender, location of onset, exact high ligation, peritoneal relaxation of the posterior wall of hernia, loss of ligation line of hernia sac, the misligation of external oblique fascia, giant hernia, ring ligation, and early getting out of bed after the operation. Assignment of the independent variable: male: yes is assigned as “1,” no is assigned as “0”; bilateral onset: yes is assigned as “1,” no is assigned as “0”; exact high ligation: yes is assigned as “1,” and no is assigned as “0”; peritoneal relaxation of posterior hernia wall: yes is assigned as “1,” and no is assigned as “0”; hernia sac ligation line falls off: yes is assigned as “1,” and no is assigned as “0”; false ligation of external oblique abdominal fascia: yes is assigned as “1,” and no is assigned as “0”; large hernia: yes is assigned as “1,” and no is assigned as “0”; banding: yes is assigned as “1,” and no is assigned as “0”; get out of bed too early after operation: yes is assigned as “1,” and no is assigned as “0.” Taking the recurrence of children after transumbilical single-site laparoscopic surgery as the dependent variable, the value of recurrence is “1,” and the value of no recurrence is “0.” The results of multiple logistic regression analysis show that male, bilateral onset, peritoneal relaxation of hernia posterior wall, detachment of hernia sac ligation line, misligation of external oblique muscle fascia, giant hernia, and early out of bed activity are the risk factors for recurrence after laparoscopic surgery in children with an indirect inguinal hernia (OR>1, *P* < 0.05); the exact high ligation and cerclage were the protective factors of recurrence (OR  <1, *P* < 0.05). The results are shown in Tables 3 and 4.

## 4. Discussions

The treatment of indirect inguinal hernia in children is less difficult than that in adult patients. Because children usually do not have weak areas of the front or back wall of the inguinal canal, most of them do not need to be repaired, and the treatment principle is to close the open sheath-like protrusion [7]. In the past, open surgery was used to treat the indirect inguinal hernia. There are many ways to open the external oblique muscle aponeurosis, high ligation of the hernia sac, and reconstruction of the outer ring. The effect is definite [8]. However, the traditional open surgery to treat an indirect inguinal hernia is very traumatic, especially for male children, which can be complicated by swelling of the affected scrotum and groin area after surgery, causing severe local pain. Because of the immature physical and mental development of children, the body's pain and trauma are poorly tolerated, and the postoperative recovery time is long; in addition, in order to avoid recurrence after traditional open surgery, it is often necessary to fully repair the incised inguinal canal of the child. The implementation of this inguinal canal repair will be effective. The children with the indirect inguinal hernia after surgery may cause secondary injuries and increase the traumatic nature of the operation [9, 10]. It can be seen that its application is limited.

Laparoscopic surgery is a minimally invasive surgical procedure that is used in many diseases, and it is also common in the treatment of inguinal hernias. Laparoscopic surgery is used for the treatment of indirect inguinal hernia. The incision made during the operation is small. After further high ligation of the hernia, the curative effect is similar to that of traditional laparotomy, the surgical trauma is smaller than traditional laparotomy, and the child can be restored better and faster after surgery [11]. The literature [12] confirmed that after laparoscopic surgery is given to children with inguinal hernia, the postoperative recurrence rate is still unsatisfactory, reaching 2.78% to 3.63%. This study performed transumbilical single-site laparoscopic surgery on 400 children with an indirect inguinal hernia, and the postoperative recurrence rate was 5.75%, which was higher than the results of the above studies. The reason for this difference may be related to the sample size and use of each study. The procedure is related to the different ages of the patients. It can be seen that children with an indirect inguinal hernia still have a higher recurrence rate after minimally invasive surgery. Single-site laparoscopic surgery through the umbilical has more advantages than conventional laparoscopic surgery, resulting in fewer traumas and less obvious scars. The postoperative recovery is faster, but the risk of recurrence is still higher. Therefore, it is particularly necessary to investigate the factors that may affect the recurrence of children with indirect inguinal hernia.

This study analyzed a variety of factors and found that older age was a high-risk factor for postoperative recurrence, mainly in the groin of younger children. The muscle tissue in this area is weak, and the hernia sac ligation process will not lead to greater tension; however, the muscle tissue develops and becomes strong with age, so it is easy to produce greater resistance during ligation, so it is likely that the hernia sac will not tighten, leading to recurrence. Through univariate and multiple logistic regression analyses, it was found that male, bilateral onset, peritoneal relaxation of the posterior wall of the hernia, loss of the ligation line of the hernia sac, misligation of the external oblique fascia, huge hernia, and early getting out of bed after operation were the risk factors for recurrence after transumbilical laparoscopic surgery in children with indirect inguinal hernia. The relationship between these factors and recurrence was analyzed as follows: (1) Male children are at risk of scrotal edema and spermatic edema on the affected side after surgery. Once the above complications are combined, the incision recovery will be delayed and the risk of recurrence will increase. (2) Bilateral onset suggests that the child's condition is serious, and laparoscopic surgery is performed to treat it. It is difficult to effectively reduce under direct vision. Poor reduction, suture, and cerclage may occur, which will increase the risk of postoperative recurrence. (3) The peritoneum of the posterior wall of the hernia can increase the difficulty of high-position ligation. The normal passage of the hernia is relatively occlusive and narrow. (4) Loss of the hernia sac ligation thread can cause ligation failure. The hernia sac can fall off and return to the original place to form a prolapsed peritoneal wall. After surgery, the resistance of the abdominal wall is weak, and the hernia block can enter the hernia sac and then increase the operation. Recurrence may occur later [13]. (5) Mistaken ligation of the external oblique fascia may be related to the size of the hernia sac. At this time, the operator may treat the external oblique fascia as a hernia sac. Increase the recurrence rate after surgery. (6) The condition of children with a giant hernia is more serious, and the diameter of the hernia block and outer ring mouth is large. It is usually necessary to repair the anterior wall of the inguinal canal. The implementation of repair will affect the progress of postoperative recovery, prolong the postoperative recovery time, and then increase the risk of recurrence. (7) Getting out of bed prematurely after surgery can cause the intra-abdominal pressure to rise to varying degrees.

After the intra-abdominal pressure rises, the hernia belt is compressed. When it is compressed below the inner ring orifice, the hernia mass cannot enter the inguinal canal through the normal passage or the scrotum, which protrudes into the abdominal wall tissue, which in turn leads to the recurrence of the child after surgery. In addition to the risk factors for recurrence obtained from the results, this study also found that exact high ligation and cerclage are the protective factors for recurrence after laparoscopic single-site laparoscopic surgery in children with indirect inguinal hernia. The main reasons are as follows: it is related to factors such as inexperienced doctors, difficulty in peeling off the hernia sac or too small hernia sac, and clear implementation of high ligation that can cure the hernia and make the contents difficult to escape, so it has a positive significance in preventing recurrence [14]. When the needle is sutured, the wall of the hernia sac may be tight, which is easy to cause longitudinal fissures, the ligation stability is poor, and the ligation thread is likely to fall off. The use of cerclage can make up for the lack of sutures. It can be sutured according to the anatomical position. It causes less damage, and the ligation is more stable, which helps prevent the recurrence of indirect inguinal hernia. Recommendations are given for the above-mentioned risk factors and protective factors for recurrence. When performing transumbilical single-site laparoscopic surgery for children with indirect inguinal hernia, a highly qualified doctor should perform the surgery and clearly grasp the child's anatomical information before surgery. Children with small hernia sacs can bluntly separate the spermatic cord, free and ligate the white membranous sheath-like process, and give the child an accurate high-position ligation according to the situation or use cerclage with a 2–0 care line; for males in children and children with bilateral disease, CT, B-ultrasound, and other methods should be used before surgery to clarify the disease and develop a targeted surgical plan; for children with huge hernia, medial umbilical fold coverage, transverse abdominal fascia repair, laparoscopic inguinal hernia repair, and autologous abdominal wall skin graft repair are feasible. After the operation, the children are guided to rest in bed and avoid getting out of bed early to reduce recurrence [15, 16]. Xuan et al. [17] and Cao and Wang. [18] pointed out that the diameter of the inner ring orifice and the use of absorbable thread are also important factors affecting the recurrence of indirect inguinal hernia in children after surgery, but this factor was not carried out in this study. The discussion and conclusions still have limitations. In the future, the research indicators and sample size should be increased to further analyze the factors affecting the recurrence of pediatric indirect inguinal hernia after laparoscopic surgery.

## 5. Conclusions

In conclusion, the recurrence of indirect inguinal hernia in children after transumbilical single-site laparoscopic surgery is affected by many factors, such as gender, location of onset, exact high ligation, relaxation of peritoneum in the posterior wall of hernia, loss of ligation line of the hernia sac, misligation of external oblique fascia, huge hernia, ring ligation, and early out of bed activities after the operation. Early evaluation of the risk of postoperative recurrence in children can be considered. Targeted intervention programs are formulated for children with high-risk factors and further improve the surgical operation to prevent the recurrence.

## Figures and Tables

**Table 1:** Univariate analysis of recurrence in children with indirect inguinal hernia after laparoscopic surgery on a single site through the umbilical surgery (case (%)).

Group	Number of cases	Age (years)			Gender		Course of disease	
		<5	6∼10	>10	Male	Female	<1	≥1
Relapse group	23	6 (26.09)	5 (21.74)	7 (52.17)	21 (91.30)	2 (8.69)	14 (60.87)	9 (39.13)
No recurrence group	377	126 (33.42)	91 (24.14)	160 (42.44)	237 (63.67)	140 (37.14)	230 (61.00)	95 (38.99)
*χ* ^2^ value		0.162			5.494		0.009	
*P* value		0.922			0.019		0.925	

**Table 2:** Univariate analysis of recurrence in children with indirect inguinal hernia after laparoscopic surgery on a single site through the umbilical surgery (case (%)).

Group	Number of cases	Disease site		High ligation		Laxation of the peritoneum on the posterior wall of the hernia		Hernia sac ligation thread falls off		Abdominal oblique muscle fascia accidentally ligated		Giant hernia		Suture or cerclage		Get out of bed prematurely after surgery	
		Unilateral	Bilateral	Yes	No	Yes	No	Yes	No	Suture	cerclage	Yes	No	Yes	No	Yes	No
Relapse group	23	9 (39.13)	14 (60.87)	8 (34.78)	15 (65.22)	9 (39.13)	14 (60.87)	11 (47.82)	12 (52.17)	14 (60.87)	9 (39.13)	8 (34.78)	15 (65.22)	17 (73.91)	6 (26.09)	9 (39.13)	14 (60.87)
No recurrence group	377	301 (79.84)	51 (20.16)	237 (63.67)	140 (37.14)	21 (9.02)	343 (90.98)	55 (14.59)	322 (85.41)	95 (25.20)	282 (74.80)	48 (12.73)	214 (87.27)	158 (41. 91)	219 (58.09)	51 (13.52)	326 (86.47)
*χ* ^2^ value		10.118		5.69		5.622		5.861		7.075		8.28		6.912		4.953	
*P* value		0.001		0.017		0.018		0.005		0.002		0.001		0.003		0.008	

**Table 3:** Multivariate logistic regression analysis results of recurrence in children with indirect inguinal hernia after laparoscopic single-site umbilical surgery.

Wald value	95% CI	Factor	*B*	S.E. value	*P* value	OR value
Male	2.078	1.044	3.964	0.046	7.987	1.033∼61.758
Bilateral onset	1.741	0.550	10.024	0.002	5.706	1.941∼16.769
Exact high ligation	1.272	0.564	5.093	0.024	0.093∼0.846	0.280
Laxation of the peritoneum on the posterior wall of the hernia	1.333	0.598	4.966	0.026	3.791	1.174∼12.242
Hernia sac ligation thread falls off	1.455	0.559	6.764	0.009	4.283	1.431∼12.817
Abdominal oblique muscle fascia accidentally ligated	1.674	0.593	7.959	0.005	5.333	1.667∼17.064
Giant hernia	1.625	0.548	8.793	0.003	5.080	1.735∼14.873
Cerclage	1.488	0.547	7.394	0.007	0.077∼0.660	0.226
Get out of bed prematurely after surgery	1.239	0.580	4.555	0.033	3.452	1.106∼10.767

**Table 4:** Multifactor influence after operation.

Influencing factors	*β*	S.E.	Wald	OR	95%CI	*P*
Age	1.56	0.45	19.54	8.61	3.41–11.69	0.00
Type of ligature	1.69	0.58	11.35	5.91	1.98–13.91	0.01
Inner ring mouth diameter	2.01	0.69	8.61	9.54	1.68–36.51	0.00

## Data Availability

The simulation experiment data used to support the findings of this study are available from the corresponding author upon request.
